The article "Anatomic Risk Factors for Osteochondral Fracture of Acute First-Time Patellar Dislocation in Adolescents: A Retrospective Magnetic Resonance Imaging Study" was retracted in 2023. Reasons: suspected computer-generated content; unreliable results or conclusions; lack of ethics approval or compliance; missing or withdrawn patient consent.

# Anatomic Risk Factors for Osteochondral Fracture of Acute First-Time Patellar Dislocation in Adolescents: A Retrospective Magnetic Resonance Imaging Study

**DOI:** 10.1155/2022/6723326

**Published:** 2022-08-08

**Authors:** Junran Li, Chuanjie Chen, Hongyan Zhou, Jingxiu Zhai, Hongbo Zhao, Ligeng Li

**Affiliations:** ^1^Department of Orthopedic Surgery, Second Hospital of Tangshan, Tangshan 063000, Hebei, China; ^2^Institute of Trauma Surgery, Second Hospital of Tangshan, Tangshan 063000, Hebei, China; ^3^Department of Orthopedic Surgery, Chengde Central Hospital, Chengde 067000, Hebei, China

## Abstract

**Objective:**

To analyze the risk factors for osteochondral fracture (OCF) of first-time acute patellar dislocation (APD) through measurements of patellofemoral anatomy in adolescents.

**Methods:**

In this prospective study, all patients were divided into two groups according to whether OCF was detected on magnetic resonance imaging (MRI): Group A (associated with OCF) and Group B (without OCF). Patellofemoral anatomy was evaluated with four aspects including trochlear/patellar dysplasia, patella location, patellofemoral matching, and morphologic classification. On MRI scans, trochlear facet asymmetry ratio (TFAR), lateral trochlear inclination (LTI), sulcus angle (SA), trochlear depth (TD), and patellar depth (PD) were measured to assess trochlear/patellar dysplasia. Insall–Salvati index (ISI), Caton–Deschamps index (CDI), Blackburne–Peel index (BPI), lateral patellofemoral angle (LPFA), patellar tilt angle (PTA), and lateral patellar displacement (LPD) were measured to show the location of patella. Patellofemoral matching was analyzed through the measurements of patellofemoral congruence angle (PFCA), patellofemoral index (PFI), and patellotrochlear index (PTI).

**Results:**

A total of ninety-four adolescents from 49 boys and 45 girls (mean age, 15 years; range, 10–18 years) with first-time APD were recruited and included in Group A (65) and Group B (29). The PFI (2.62 ± 0.51 *vs*. 2.10 ± 0.44) and PTI (0.28 ± 0.05 *vs*. 0.22 ± 0.07) were significantly higher in Group B than Group A (*P* < 0.05). There were no significant differences in other quantitative outcomes of the two groups (*P* > 0.05). The distribution of Dejour/Wiberg classification was statistically similar between the two groups (*P* > 0.05).

**Conclusions:**

Adolescent patients with first-time APD complicating OCF have closer morphologic features of patellofemoral dysplasia and patella location when compared to adolescents without OCF. Abnormal patellofemoral matching increases the risk of OCF after first-time APD in adolescents.

## 1. Introduction

Acute patellar dislocation (APD) is a clinically common injury, especially in adolescents [1]. Recent epidemiologic studies show that the annual risk for first-time patellar dislocation among 10 to 17-year-old populations is approximately 29 per 100,000 [2]. Most patients who experience a patellar dislocation usually have concomitant injuries of medial patellofemoral ligament (MPFL) and cartilage after the transient displacement and reduction [3, 4]. MPFL tears can be confirmed by physical examination and radiographic evaluation. However, omission diagnosis for the loose body in this lesion could take place because the location, extent, and frequency of the osteochondral fracture (OCF) fragments are various [3]. Although large fragments may be found on plain radiographs, smaller fragments which only contained a slice of subcartilaginous bone may become unrecognized. If left untreated in time, chondral defects result in persistent pain, daily activity limitation, and may generate traumatic arthritis in the future. Increasing diagnostic accuracy of OCF is necessary to establish an appropriate treatment [5].

The article "Anatomic Risk Factors for Osteochondral Fracture of Acute First-Time Patellar Dislocation in Adolescents: A Retrospective Magnetic Resonance Imaging Study" was retracted in 2023. Reasons: suspected computer-generated content; unreliable results or conclusions; lack of ethics approval or compliance; missing or withdrawn patient consent.

Magnetic resonance imaging (MRI) is an irreplaceable diagnostic examination in delineating the structural features of soft tissues for knee joint [6]. Pathoanatomical factors (e.g., trochlear/patellar dysplasia, patella alta, and malalignment syndromes) assessed on MRI predisposing to APD have been demonstrated in many clinical reports [7, 8]. Nevertheless, previous studies based on the anatomic risk factors for APD with OCF are scarce. OCF may be associated with some anatomical malformations, and the implications of this event on clinical practice are unclear. Unfortunately, redislocation rate of APD ranges from 10 to 26% after surgical treatment [9, 10]. In other words, children and adolescents with first-time APD have a high probability of secondary patellar dislocation with OCF after initial operation. Therefore, treatment algorithm should be individualized based on the both injury and deformity.

The purpose of this study was to analyze potential anatomic risk factors leading to first-time APD complicating OCF in adolescent populations. We hypothesized that our study findings could reveal some classic anatomic parameters that might relate to OCF. It could also provide better understanding of injury mechanism and theoretical guidance for accurate diagnosis.

## 2. Materials and Methods

### 2.1. Subjects

This retrospective study included consecutive patients with first-time APD who had undergone hospitalization from 2011 through 2020 and was approved by the required institutional review boards of level-I trauma centers (No. TSEY-LL-L20220013). All patients were divided into two groups according to the diagnosis of OCF: Group A (first-time APD children with OCF) and Group B (without OCF).

The article "Anatomic Risk Factors for Osteochondral Fracture of Acute First-Time Patellar Dislocation in Adolescents: A Retrospective Magnetic Resonance Imaging Study" was retracted in 2023. Reasons: suspected computer-generated content; unreliable results or conclusions; lack of ethics approval or compliance; missing or withdrawn patient consent.

### 2.2. Inclusion Criteria and Exclusion Criteria

The inclusion criteria for this study were defined as follows: ① age 18 years or younger; ② first-time APD was diagnosed based on MRI [11]; and ③ presentation less than 3 weeks from injury. The exclusion criteria were as follows: ① patients who were suspected to have the history of operation or trauma; ② patients without MRI data or insufficient quality; ③ medial patellar dislocation; and ④ preexisting ipsilateral knee diseases (Charcot arthritis, rheumatoid arthritis, and so on).

## 3. Methods

The MRI was performed on a GE 1.5 Tesla magnet. The sequences were obtained as follows: sagittal T1-weighted image (T1WI) views were achieved by using a spin echo sequence system, while sagittal T2-weighted image (T2WI) views were obtained by a fast spin echo sequence system. Slice thickness was 3 mm with 1 mm gap, and sequence parameters were repetition time (TR) of 1892 ms/echo time (TE) of 10.1 ms for T1WI and TR of 2700 ms /TE of 123 ms for T2WI.

All imaging data were identified from the picture archiving and communication system (PACS). The MRI scans were evaluated for all cases, and the anatomic parameters were measured blindly by two trained orthopedists who specialized in pediatric sports medicine. To minimize errors, the mean value of measurements for each parameter was recorded.

### 3.1. Observational Indicators

#### 3.1.1. Trochlear/Patellar Dysplasia

Trochlear facet asymmetry ratio (TFAR), lateral trochlear inclination (LTI), sulcus angle (SA), trochlear depth (TD), and patellar depth (PD) were measured to assess trochlear or patellar dysplasia on axial knee MRI [12–15].

#### 3.1.2. Patella Location

Patellar height (vertical location) was assessed by using the Insall–Salvati index (ISI), Caton–Deschamps index (CDI), and Blackburne–Peel index (BPI) on sagittal knee MRI at the midsagittal slice [16–18]. Patella horizontal location was assessed by lateral patellofemoral angle (LPFA), patellar tilt angle (PTA), and lateral patellar displacement (LPD) on axial scan [19–21].

#### 3.1.3. Patellofemoral Matching

Patellofemoral congruence angle (PFCA), patellofemoral index (PFI), and patellotrochlear index (PTI) were measured to assess the matching of patellofemoral joint [22, 23].

#### 3.1.4. Trochlear/Patellar Classification

The morphology of dysplastic trochlea and patella were evaluated by Dejour classification and Wiberg classification [24, 25], respectively.

### 3.2. Statistical Analysis

All statistical data in our study were analyzed with SPSS 25.0 software (IBM, Armonk, New York, USA). Continuous variables were used to analyze and presented as mean ± standard deviation. According to whether the variables conformed to a normal distribution, the independent *t*-test or Mann–Whitney *U* test was used for the comparison of continuous variables. Differences in categorical variables were compared using the chi-square test or Fisher's exact test. A *P* value of <0.05 was considered as statistically significant.

The article "Anatomic Risk Factors for Osteochondral Fracture of Acute First-Time Patellar Dislocation in Adolescents: A Retrospective Magnetic Resonance Imaging Study" was retracted in 2023. Reasons: suspected computer-generated content; unreliable results or conclusions; lack of ethics approval or compliance; missing or withdrawn patient consent.

## 4. Results

One ninety-four (49 boys and 45 girls) MRI scans were reviewed, with a mean age of 15 years (range, 10–18 years). Sixty-five adolescents were allocated into Group A (associated OCF), and twenty-nine adolescents were allocated into Group B (without OCF). Patient demographics of two groups are summarized, as shown in Table 1. The mean age, the gender distribution, and other baseline features were statistically similar between two groups (*P* > 0.05).

All measured results of anatomic parameters for trochlear/patellar dysplasia, patella location, and patellofemoral matching are provided in Tables 2–4, respectively. The PFI and PTI of Group B were (2.62 ± 0.51 and 0.28 ± 0.05), which were significantly higher than those of Group A (2.10 ± 0.44 and 0.22 ± 0.07) (*P* < 0.05). There was no statistically significant difference between TFAR, LTI, SA, TD, PD, ISI, CDI, BPI, LPFA, PTA, LPD, and PFCA of the two groups (*P* > 0.05). No significant differences were observed in the distribution of Dejour and Wiberg classification between the two groups (*P* > 0.05), as shown in Table 5.

## 5. Discussion

APD is a common spontaneous knee injury and tends to occur in adolescent active population [1, 26]. It is mainly because of patellofemoral bony malformations and imbalanced soft tissue [27]. Eventually, the patella goes out of control from normal trajectory and displaces to the lateral position. Meanwhile, a direct blow from the medial patella to lateral femoral condyle usually results in OCF [3, 4]. In this study, we combined some qualitative and quantitative outcomes to assess anatomic factors for first-time APD in adolescents. The findings in this study were that the occurrence of OCF was related to PFI and PTI. Patella location and morphology of trochlea/patella might not increase the risk of OCF.

The patella has a physiological tendency to slide laterally when the knee keeps flexion over enough angles [28]. The innate patellofemoral apparatus provides a stability to maintain a normal moving trajectory and prevents lateral displacement of the patella. Well-balanced soft tissue system contributes to dynamic stability [29], and it is composed of four components from different directions just like a perpendicular cross: proximal side is quadriceps femoris; distal side is patellar ligament; medial side includes MPFL, medial retinaculum, and medial vastus muscle; lateral side includes vastus lateralis muscle, lateral retinaculum, and iliotibial tract. As people get older, the dynamic strength of inhibition could be changed to adapt bone growth and sports activity.

The article "Anatomic Risk Factors for Osteochondral Fracture of Acute First-Time Patellar Dislocation in Adolescents: A Retrospective Magnetic Resonance Imaging Study" was retracted in 2023. Reasons: suspected computer-generated content; unreliable results or conclusions; lack of ethics approval or compliance; missing or withdrawn patient consent.

The static strength of inhibition mainly originated from patellofemoral bony structure (femoral trochlea and articular surface of patella). Over the past years, many scholars [30–32] reported that anatomic abnormalities of the patella and femoral trochlea were independent risk factors for APD. So theoretically, pathoanatomical parameters of patellofemoral joint may aggravate the trend of APD and then lead to OCF with a great possibility. From the measuring results of trochlear and patellar morphology, we found that TFAR, LTI, SA, TD, and PD remained abnormal from both groups and there was no statistical difference between two groups. This means trochlear or patellar dysplasia may not play a role to provide a strong blow, resulting in OCF. After treating OCF by surgeons, osteoplasty of trochlear groove or patellar surface needs to be considered carefully. Perhaps there are no benefits to prognosis outcomes.

We evaluated the position of the patella in our study population, recording anatomic parameters on both sagittal and axial views. For sagittal views, patella alta was regarded as a risk factor for lateral patellar instability, and the incidence of patella alta in first-time APD was approximately 25% [8]. In this series, we found no difference in ISI, CDI, and BPI between two groups. This finding demonstrated that patellar height was not the cause of OCF. For axial views, MPFL is the primary ligamentous restraint to lateral patellar stability. Elias et al. [33] reported in their study that 49% of patients with APD were accompanied by MPFL injury. Previous studies for adolescents also have shown a high incidence of injury to the MPFL on MRI in first-time APD [34, 35]. Repair or reconstruction of the MPFL after APD is controversial for adolescents. However, if a child is undergoing the operation for OCF, addressing the medial structures concomitantly might spare the patient recurrence and subsequent operations. Seeley et al. [36] undertook MPFL and OCF repair at the time of surgery, and the follow-up results turned out to be satisfactory. In the study, there was no statistical difference of LPFA, PTA, and LDP between Group A and Group B, indicating that axial linear patellar displacement was not associated with the occurrence of OCF. Even so, our study found that loose or torn MPFL and other injured soft tissues can lead to the decreased ligament strength. The patella was able to displace variably in many placements even leaving from the trochlear groove. Ultimately, inevitable measured errors would occur for assessment of axial patellar displacement. Further anatomical studies could be established to create a new measuring method to solve this problem.

The article "Anatomic Risk Factors for Osteochondral Fracture of Acute First-Time Patellar Dislocation in Adolescents: A Retrospective Magnetic Resonance Imaging Study" was retracted in 2023. Reasons: suspected computer-generated content; unreliable results or conclusions; lack of ethics approval or compliance; missing or withdrawn patient consent.

In this study, the results of measurements showed that PFI and PTI of Group B were significantly higher than those in Group A. PFI and PTI not only predisposed to patellofemoral joint instability but also contributed to OCF risk. In brief, we found that abnormal patellofemoral matching may increase risk of OCF after first-time APD. Uimonen et al. [37], studying the risk of OCF after APD, also pointed out that bony malformations and patella location may not increase risk of OCF, and PFI and PTI values were worth recommended in practice. Anatomically, the trochlear groove is concave, whereas the articular surface of the patella is convex. During the time of transient dislocation, similar medial and lateral patellofemoral joint space leads to time delay of impact from the patella to lateral femoral condyle, and impact points were located at the patellar crest, so does the mechanism of relocation: the contact area between the lateral femur and the patellar crest is reduced, and the resistance is more concentrated, resulting in a corresponding increase in local pressure. It may be in part account for the higher incidence of osteochondral injury. However, no significant difference was found in PFCA for group comparison. The measurements of PFCA are affected by SA and patella horizontal location. During the processes of dislocation and relocation, flexible location of the patella may also affect the results of the measurement.

The strengths of this study included the comprehensive anatomical measurements, and common injury pattern of OCF after APD was analyzed. Furthermore, measuring results for adolescents were conducted by two trained observers, which effectually improved the reliability of the measurements. The current study had some limitations. First, the sample size was small. Some patients with no or insufficient MRI were not included, which might have limited the generalizability of the study results. Second, all results were measured after dislocation and relocation, leading to the direction and distance of the displaced patella being changed, which could cause inevitable errors for a part of parameters. Third, the occurrence of OCF was a multifactorial consequence. More anatomical factors, such as soft tissue factors, could be evaluated under a further study.

In conclusion, first-time APD with OCF remains a common injury pattern in adolescent patients. The adolescents with or without OCF have closer trochlear/patellar dysplastic morphology and patella location. Patellofemoral matched malformation may contribute to the risk of OCF in this injury pattern.

The article "Anatomic Risk Factors for Osteochondral Fracture of Acute First-Time Patellar Dislocation in Adolescents: A Retrospective Magnetic Resonance Imaging Study" was retracted in 2023. Reasons: suspected computer-generated content; unreliable results or conclusions; lack of ethics approval or compliance; missing or withdrawn patient consent.

## Figures and Tables

**Table 1:** Comparison of demographics between two groups.

Variable	Group A (*n* = 65)	Group B (*n* = 29)	*P* value
Mean age, years	15.14 ± 2.04	14.59 ± 2.04	0.228
Gender, *n* (%)			0.164
Boy	37 (56.9%)	12 (41.4%)	
Girl	28 (43.1%)	17 (58.6%)	
Side of injury, *n* (%)			0.545
Left	29 (44.6%)	11 (37.9%)	
Right	36 (55.4%)	18 (62.1%)	
Injury reason, *n* (%)			0.726
Sports	37 (56.9%)	14 (48.3%)	
Daily activity	16 (24.6%)	9 (31.0%)	
Unknown	12 (18.5%)	6 (20.7%)	
First-time APD to MRI time (days)	8.43 ± 4.53	6.97 ± 3.70	0.130

**Table 2:** Comparison of trochlear/patellar dysplastic parameters between two groups.

	Group A (*n* = 65)	Group B (*n* = 29)	*P* value
Trochlear facet asymmetry ratio	0.51 ± 0.10	0.49 ± 0.11	0.427
Lateral trochlear inclination (°)	14.22 ± 2.11	13.60 ± 2.17	0.175
Sulcus angle (°)	153.82 ± 7.72	152.13 ± 9.75	0.489
Trochlear depth (mm)	2.09 ± 0.84	2.16 ± 0.76	0.703
Patellar depth (mm)	3.93 ± 0.44	3.83 ± 0.49	0.374

**Table 3:** Comparison of patella location between two groups.

	Group A (*n* = 65)	Group B (*n* = 29)	*P* value
Insall–Salvati index	1.28 ± 0.18	1.25 ± 0.18	0.429
Caton–Deschamps index	1.22 ± 0.19	1.18 ± 0.16	0.260
Blackburne–Peel index	1.09 ± 0.22	1.07 ± 0.15	0.338
Lateral patellofemoral angle (°)	15.40 ± 3.91	14.74 ± 4.92	0.545
Patellar tilt angle (°)	19.05 ± 5.66	18.21 ± 6.08	0.284
Lateral patellar displacement (mm)	13.76 ± 4.54	14.28 ± 4.63	0.615

**Table 4:** Comparison of patellofemoral matching between two groups.

	Group A (*n* = 65)	Group B (*n* = 29)	*P* value
Patellofemoral congruence angle (°)	27.34 ± 10.21	25.53 ± 9.47	0.523
Patellofemoral index	2.10 ± 0.44	2.62 ± 0.51	<0.001
Patellotrochlear index	0.22 ± 0.07	0.28 ± 0.05	<0.001

**Table 5:** The morphologic classification of dysplastic trochlea and patella.

	Group A (*n* = 65)	Group B (*n* = 29)	*P* value
Dejour classification			0.597
Type I	32	10	
Type II	11	6	
Type III	13	7	
Type IV	9	6	

Wiberg classification			0.319
Type I	9	6	
Type II	16	10	
Type III	40	13	

## Data Availability

The data used during the present study are available from the corresponding author upon request.

## References

[1] Schneider D. K., Grawe B., Magnussen R. A. (2016). Outcomes after isolated medial patellofemoral ligament reconstruction for the treatment of recurrent lateral patellar dislocations: a systematic review and meta-analysis. *The American Journal of Sports Medicine*.

[2] Fithian D. C., Paxton E. W., Stone M. L. (2004). Epidemiology and natural history of acute patellar dislocation. *The American Journal of Sports Medicine*.

The article "Anatomic Risk Factors for Osteochondral Fracture of Acute First-Time Patellar Dislocation in Adolescents: A Retrospective Magnetic Resonance Imaging Study" was retracted in 2023. Reasons: suspected computer-generated content; unreliable results or conclusions; lack of ethics approval or compliance; missing or withdrawn patient consent.

[3] Martin N. J., Lustig S., Servien E., Mangiavini L., Luceri F. (2020). Transosseous suture loop technique for MPFL reconstruction. *Journal of Biological Regulators & Homeostatic Agents*.

[4] Bauer K. L. (2018). Osteochondral injuries of the knee in pediatric patients. *Journal of Knee Surgery*.

[5] Nomura E., Inoue M. (2005). Second-look arthroscopy of cartilage changes of the patellofemoral joint, especially the patella, following acute and recurrent patellar dislocation. *Osteoarthritis and Cartilage*.

[6] Askenberger M., Arendt E. A., Ekström W., Voss U., Finnbogason T., Janarv P. M. (2016). Medial patellofemoral ligament injuries in children with first-time lateral patellar dislocations: a magnetic resonance imaging and arthroscopic study. *The American Journal of Sports Medicine*.

[7] Migliorini F., Maffulli N., Eschweiler J., Quack V., Tingart M., Driessen A. (2021). Lateral retinacular release combined with MPFL reconstruction for patellofemoral instability: a systematic review. *Archives of Orthopaedic and Trauma Surgery*.

[8] Balcarek P., Ammon J., Frosch S. (2010). Magnetic resonance imaging characteristics of the medial patellofemoral ligament lesion in acute lateral patellar dislocations considering trochlear dysplasia, patella alta, and tibial tuberosity-trochlear groove distance. *Arthroscopy: The Journal of Arthroscopic & Related Surgery*.

[9] Smith T. O., Donell S., Song F., Hing C. B. (2015). Surgical versus non-surgical interventions for treating patellar dislocation. *Cochrane Database of Systematic Reviews*.

[10] Cheng B., Wu X., Ge H., Qing Sun Y., Zhang Q. (2014). Operative versus conservative treatment for patellar dislocation: a meta-analysis of 7 randomized controlled trials. *Diagnostic Pathology*.

[11] Sillanpää P., Mattila V. M., Iivonen T., Visuri T., Pihlajamäki H. (2008). Incidence and risk factors of acute traumatic primary patellar dislocation. *Medicine & Science in Sports & Exercise*.

[12] Pfirrmann C. W. A., Zanetti M., Romero J., Hodler J. (2000). Femoral trochlear dysplasia: MR findings. *Radiology*.

[13] Brattström H. (1964). Shape of the intercondylar groove normally and in recurrent dislocation of patella. a clinical and x-ray-anatomical investigation. *Acta Orthopaedica Scandinavica*.

[14] Paiva M., Blønd L., Hölmich P. (2018). Quality assessment of radiological measurements of trochlear dysplasia; a literature review. *Knee Surgery, Sports Traumatology, Arthroscopy*.

[15] Biedert R. M., Bachmann M. (2009). Anterior-posterior trochlear measurements of normal and dysplastic trochlea by axial magnetic resonance imaging. *Knee Surgery, Sports Traumatology, Arthroscopy*.

The article "Anatomic Risk Factors for Osteochondral Fracture of Acute First-Time Patellar Dislocation in Adolescents: A Retrospective Magnetic Resonance Imaging Study" was retracted in 2023. Reasons: suspected computer-generated content; unreliable results or conclusions; lack of ethics approval or compliance; missing or withdrawn patient consent.

[16] Caton J. H., Prudhon J. L., Aslanian T., Verdier R. (2016). Patellar height assessment in total knee arthroplasty: a new method. *International Orthopaedics*.

[17] Blackburne J. S., Peel T. E. (1977). A new method of measuring patellar height. *Journal of Bone and Joint Surgery British Volume*.

[18] Insall J., Salvati E. (1971). Patella position in the normal knee joint. *Radiology*.

[19] Laurin C. A., Lévesque H. P., Dussault R., Labelle H., Peides J. P. (1978). The abnormal lateral patellofemoral angle: a diagnostic roentgenographic sign of recurrent patellar subluxation. *The Journal of Bone and Joint Surgery*.

[20] Grelsamer R. P., Bazos A. N., Proctor C. S. (1993). Radiographic analysis of patellar tilt. *Journal of Bone and Joint Surgery British Volume*.

[21] Urch S. E., Tritle B. A., Donald Shelbourne K., Gray T. (2009). Axial linear patellar displacement: a new measurement of patellofemoral congruence. *The American Journal of Sports Medicine*.

[22] Lankhorst N. E., Bierma-Zeinstra S. M. A., van Middelkoop M. (2013). Factors associated with patellofemoral pain syndrome: a systematic review. *British Journal of Sports Medicine*.

[23] Yuksel Y., Ergun T., Torun E., Unal M., Sonnow L., Kose O. (2021). The relationship between quadriceps fat pad syndrome and patellofemoral morphology: a case-control study. *Journal of Orthopaedics and Traumatology*.

[24] Dejour D., Le Coultre B. (2018). Osteotomies in patello-femoral instabilities. *Sports Medicine and Arthroscopy Review*.

[25] Aksu N., Atansay V., Karalök I., Aksu T., Kara A. N., Hamzaoglu A. (2021). Relationship of patellofemoral angles and tibiofemoral rotational angles with jumper’s knee in professional dancers: an MRI analysis. *Orthopaedic Journal of Sports Medicine*.

[26] Antinolfi P., Bartoli M., Placella G. (2016). Acute patellofemoral instability in children and adolescents. *Joints*.

[27] Hartmann F., Dietz S. O., Rommens P. M., Gercek E. (2014). Long-term outcome after operative treatment of traumatic patellar dislocation in adolescents. *Journal of Orthopaedic Trauma*.

[28] Zheng L., Shi H., Feng Y., Sun B. S., Ding H. Y., Zhang G. Y. (2015). Injury patterns of medial patellofemoral ligament and correlation analysis with articular cartilage lesions of the lateral femoral condyle after acute lateral patellar dislocation in children and adolescents: an MRI evaluation. *Injury*.

[29] Kang H. J., Wang F., Chen B. C., Su Y. L., Zhang Z. C., Yan C. B. (2010). Functional bundles of the medial patellofemoral ligament. *Knee Surgery, Sports Traumatology, Arthroscopy*.

The article "Anatomic Risk Factors for Osteochondral Fracture of Acute First-Time Patellar Dislocation in Adolescents: A Retrospective Magnetic Resonance Imaging Study" was retracted in 2023. Reasons: suspected computer-generated content; unreliable results or conclusions; lack of ethics approval or compliance; missing or withdrawn patient consent.

[30] Amis A. A. (2007). Current concepts on anatomy and biomechanics of patellar stability. *Sports Medicine and Arthroscopy Review*.

[31] Kita K., Tanaka Y., Toritsuka Y. (2015). Factors affecting the outcomes of double-bundle medial patellofemoral ligament reconstruction for recurrent patellar dislocations evaluated by multivariate analysis. *The American Journal of Sports Medicine*.

[32] Fucentese S. F., von Roll A., Koch P. P., Epari D. R., Fuchs B., Schottle P. B. (2006). The patella morphology in trochlear dysplasia—a comparative MRI study. *The Knee*.

[33] Elias D. A., White L. M., Fithian D. C. (2002). Acute lateral patellar dislocation at MR imaging: injury patterns of medial patellar soft-tissue restraints and osteochondral injuries of the inferomedial patella. *Radiology*.

[34] Seeley M., Bowman K. F., Walsh C., Sabb B. J., Vanderhave K. L. (2012). Magnetic resonance imaging of acute patellar dislocation in children: patterns of injury and risk factors for recurrence. *Journal of Pediatric Orthopaedics*.

[35] Kepler C. K., Bogner E. A., Hammoud S., Malcolmson G., Potter H. G., Green D. W. (2011). Zone of injury of the medial patellofemoral ligament after acute patellar dislocation in children and adolescents. *The American Journal of Sports Medicine*.

[36] Seeley M. A., Knesek M., Vanderhave K. L. (2013). Osteochondral injury after acute patellar dislocation in children and adolescents. *Journal of Pediatric Orthopaedics*.

[37] Uimonen M., Ponkilainen V., Hirvinen S. (2021). The risk of osteochondral fracture after patellar dislocation is related to patellofemoral anatomy. *Knee Surgery, Sports Traumatology, Arthroscopy*.

